The article "Application of Machine Learning Techniques to Detect the Children with Autism Spectrum Disorder" was published in 2022. Journal: J Healthc Eng.

# Application of Machine Learning Techniques to Detect the Children with Autism Spectrum Disorder

**DOI:** 10.1155/2022/9340027

**Published:** 2022-03-25

**Authors:** Mengyi Liao, Hengyao Duan, Guangshuai Wang

**Affiliations:** ^1^Department of Education, Pingdingshan University, Pingdingshan 467000, China; ^2^National Engineering Laboratory for Technology of Big Data Application in Education, Central China Normal University, Wuhan 430079, China

## Abstract

Early detection of autism spectrum disorder (ASD) is highly beneficial to the health sustainability of children. Existing detection methods depend on the assessment of experts, which are subjective and costly. In this study, we proposed a machine learning approach that fuses physiological data (electroencephalography, EEG) and behavioral data (eye fixation and facial expression) to detect children with ASD. Its implementation can improve detection efficiency and reduce costs. First, we used an innovative approach to extract features of eye fixation, facial expression, and EEG data. Then, a hybrid fusion approach based on a weighted naive Bayes algorithm was presented for multimodal data fusion with a classification accuracy of 87.50%. Results suggest that the machine learning classification approach in this study is effective for the early detection of ASD. Confusion matrices and graphs demonstrate that eye fixation, facial expression, and EEG have different discriminative powers for the detection of ASD and typically developing children, and EEG may be the most discriminative information. The physiological and behavioral data have important complementary characteristics. Thus, the machine learning approach proposed in this study, which combines the complementary information, can significantly improve classification accuracy.

## 1. Introduction

Autism spectrum disorder (ASD) is a neurological developmental disorder involving behavioral and cognitive impairment, and it usually begins in early childhood [1]. However, the cause of ASD is unclear, and no effective medical measures could be used [2]. The Centers for Disease Control and Prevention of the United States reported that the number of children diagnosed with ASD has dramatically increased over the past decade, reaching 1 in 54 in the USA [3]. ASD has become a worldwide medical problem and a tremendous economic and mental burden to society. An emerging view is that the atypical behavior of ASD children may be caused by early brain adaptation to an adverse environment, rather than a result of ongoing neural pathology [4]. Children's brains are rapidly developing in early childhood. Hence, early detection and intervention could prevent the brain adaptation to an adverse environment and significantly improve the prognosis. Previous studies have shown children's neural plasticity degeneration with increasing age, and the early intervention of children can effectively improve their language and cognitive abilities in the onset of behavioral problems [5]. Therefore, the early detection of ASD is of great significance.

Unfortunately, most ASD detection tools in use today produce diagnosis by manual observation, which are time-consuming and difficult to apply. For example, the Modified Checklist for Autism in Toddlers [6], which is a standard questionnaire for parents, is administered by specialists in rigorously controlled clinical settings, usually taking hours to complete [7]. Thus, an intelligent automatic detection tool is needed to improve detection efficiency and operability.

Many physiological and behavioral data have been demonstrated useful in ASD detection in typically developing (TD) children [8]. Children with ASD have disorders in social interaction, especially in nonverbal behaviors, such as eye contact and facial expression imitation, lacking common attention, social interaction, and emotional sharing. Considerable literature related to the study of eye fixation in children with ASD exists. For instance, Wang et al. [9] examined 31 children with ASD and 51 TD peers and asked them to scan emotional faces. The children with ASD highlighted multiple differences in gaze patterns compared with the TD children. The results suggested that fixation count, fixation duration, and average saccade velocity may be used as indicators for the early identification of ASD. Sassoon et al. [10] discovered that, when presented with social and nonsocial objects, children with ASD paid considerable attention to nonsocial objects, whereas TD children paid considerable attention to social objects. In consideration of the atypical gaze-scanning patterns in ASD, machine learning has been used to detect children with ASD. For example, Liu et al. [11] developed a machine learning algorithm based on face-scanning patterns for classification and identified children with ASD with an accuracy of 82.51%, indicating promising evidence for applying machine learning algorithms to identify children with ASD. Jiang and Francis [12] proposed a machine learning method to classify the eye fixations of ASD and TD children, which achieved a classification accuracy of 84%. These studies demonstrated that machine learning has advantages in efficiency and objectiveness compared with standardized diagnostic scales. Compared with TD children, children with ASD have disorders in nonverbal communication skills, such as the abilities of facial expression recognition (FER) and expression imitation. Samad et al. [13] evaluated the ability of ASD children to imitate others' facial expressions on the basis of their expression muscles. The results suggested that spontaneous expression imitation could be used as a behavioral marker of children with ASD. Jaiswal et al. [7] developed an algorithm that automatically detects ASD in individuals with attention-deficit hyperactivity disorder by using facial expression data based on dynamic deep learning and 3D analysis of behavior. This study found that using facial expression data to detect ASD is effective.

Atypical brain development in children with ASD appears earlier than atypical behavior, and the critical period of early intervention will be missed if the detection is based on behavioral data. This condition has fueled the research of ASD detection in the prodromal phase by using physiological data, such as electroencephalography (EEG) data. EEG was originally used to measure cortical activity in children. Owing to the advantages of noninvasiveness, low cost, and high temporal resolution, EEG has become a useful biological indicator of brain development in children [14]. Abdulhay et al. [15] proposed an EEG-based quantitative approach for the automatic detection of ASD in TD children, relying on a second-order difference plot area as a discriminative feature. Bosl et al. [16] analyzed nonlinear features of EEG signals to assist in the diagnosis of ASD with high accuracy, specificity, and sensitivity. Ibrahim et al. [17] investigated different EEG feature extraction and classification techniques to predict the clinical diagnostic outcome of epilepsy and ASD, improving the speed and accuracy of diagnosis.

Although the data of eye fixation, facial expression, and EEG have been applied to detect ASD, studies on data fusion are few, the discriminative powers of different data modalities are unclear, and the complementary characteristics of such data modalities should be investigated. In this study, we used an innovative approach to extract features of eye fixation, facial expression, and EEG, and a hybrid fusion approach based on a weighted naive Bayes algorithm was presented for multimodal data fusion. Then, confusion matrices and graphs were analyzed to investigate the complementary characteristics and discriminative powers of different data modalities. The contributions of this study are summarized as follows: (1) the limitation of single-dimensional detection is avoided by detecting ASD from two dimensions: physiology (EEG) and behavior (eye fixation and facial expression); (2) the discriminative powers of different data modalities were investigated, and EEG may be the most discriminative information compared with eye fixation and facial expression data; and (3) a hybrid fusion approach based on a weighted naive Bayes algorithm was developed to improve classification accuracy by combining the complementary information of the three modalities.

In Section 2, the data and methodology are presented. In Section 3, a feature extraction method is provided. A weighted naive Bayes algorithm is presented in Section 4, wherein the details of a hybrid fusion framework are also described. The experimental results are provided in Section 5, and the conclusions are given in Section 6.

## 2. Proposed Method

### 2.1. Data

Eighty children with and without ASD completed the study. They were recruited from special education schools and regular kindergartens. All subjects were recruited with the approval of our institutional review board. Forty children (age range: 3–6 years; mean ± SD: 4.6 ± 9 months; the number of boys: 33; the number of girls: 7) were diagnosed with ASD on the basis of the criteria of the Diagnostic and Statistical Manual of Mental Disorders, Fifth Edition. Forty TD controls (age range: 3–6 years; mean ± SD: 4.8 ± 7 months; the number of boys: 33; the number of girls: 7) were screened to exclude any with psychiatric or neurological disorders, including ASD. No significant difference in age or sex existed between the two groups of participants.

A video clip, containing social and nonsocial information, was edited as the stimulus. The social information is comedians with happy facial expressions, funny actions, and laughter. There were 10 video clips in total in our material pool, and three graduate students majoring in special education were asked to assess their emotions when watching the video clips in two dimensions (valence-arousal). The valence changes from negative to positive. The arousal dimension changes from calm to excited. The mean distributions of the 10 video clips on the arousal-valence plane were counted. The video clip with the highest mean arousal of positive was selected from the material pool. The nonsocial information includes backgrounds and two spinning wheels. The video clip lasts 40 s. Previous studies have found that children with ASD have atypical processing patterns for social information, reflected in abnormal eye fixation, facial expressions, and EEG data [18, 19]. These multimodal data were collected with three sensors, Tobii Eye Tracker, video camera, and Emotiv EPOC+. Tobii Eye Tracker was used to collect the data of eye fixation of children, a video camera was used to collect facial expressions of children, and Emotiv EPOC+ was used to collect EEG data of children. We intended to detect children with ASD by analyzing multimodal data reflecting the children's atypical processing patterns for social information.

### 2.2. Framework

In this study, a multimodal framework capable of automatically detecting children with ASD was proposed. The experimental scene and data analysis method are shown in Figure 1. Four stages were considered. (1) In the data acquisition stage, multimodal data were collected with three sensors when the children were providing the stimulus. (2) The eye fixation, facial expression, and EEG features were extracted in the feature extraction stage. (3) The behavioral features were fused with eye fixation and facial expression features, and then, the behavioral and physiological features were sent to a classification model to produce subdecisions. (4) The subdecisions were the inputs of the decision fusion, and a weighted naive Bayes algorithm was used for the final classification result.

## 3. Feature Extraction

### 3.1. Eye Fixation Features

Existing studies have shown that children with ASD have atypical social attention compared with TD children [20]. Children with ASD pay considerable attention to nonsocial information, whereas TD children pay considerable attention to social information. Data of eye fixation are the coordinate of the participants' fixation points. Therefore, we regarded fixation points as discriminative features for ASD classification. We divided the number of all fixation points by the number of fixation points in a region to produce a distribution frequency. The higher the distribution frequency is, the higher the interest in information will be. Different areas of interest (AOI) can be divided on the basis of fixation coordinates. In this study, *K*-means algorithm was used to cluster the fixation points of the participants. All the fixation points were clustered to *K* clusters, corresponding to *K* distribution frequency, which was considered *K* eye fixation feature. A binary variable *r*_*nk*_ ∈ {0,1} was introduced to represent the relationship of the fixation point *n* and cluster *K*. If fixation point *n* belongs to cluster *K*, the value of *r*_*nk*_ is 1; otherwise, it is 0. Therefore, loss function *J* can be defined as follows:

(1) $$\begin{array}{c} J=\sum_{n=1}^{N}\sum_{k=1}^{K}r_{nk}{\left\|n-\mu_{k}\right\|}^{2} \end{array}$$

where *μ*_*k*_ is the center of cluster *K*, and *J* represents the sum of squares of the distance from each fixation point to the clustering center. *K*-means performs an iterative algorithm to obtain optimal *r*_*nk*_ and *μ*_*k*_. The iterative algorithm can be described as follows:

**Step 1 .**

*r*_*nk*_ that can minimize loss function *J*, which is a linear function of *r*_*nk*_, is calculated. Given the values of *n* and *μ*_*k*_, the fixation point is assigned to the nearest cluster.

(2) $$\begin{array}{c} r_{nk}=\left\{\begin{array}{cc} 1, & k=\arg\min{\left\|n-\mu_{j}\right\|}^{2},\\ 0, & \mathrm{otherwise}\text{.} \end{array}\right. \end{array}$$

**Step 2 .**

In accordance with *r*_*nk*_, the cluster center *μ*_*k*_ that minimizes loss function *J* can be obtained. *J* is a quadratic function of *μ*_*k*_, and the following equation can be obtained when the derivative of *J* with respect to *μ*_*k*_ is 0.

(3) $$\begin{array}{c} \sum_{n=1}^{N}r_{nk}\left(x_{n}-\mu_{k}\right)=0. \end{array}$$

Hence, *μ*_*k*_ can be calculated as follows:

(4) $$\begin{array}{c} \mu_{k}=\frac{\sum_{n=1}^{N}r_{nk}x_{n}}{\sum_{n=1}^{N}r_{nk}}. \end{array}$$

Steps 1 and 2 are iterated until *μ*_*k*_ converges, and the optimal cluster center *K* can be obtained.

In our study, *K* was set to 8, 12, 16, and 20, and we divided different AOIs by using the *K*-means algorithm, as shown in Figure 2. The final value of *K* was determined from the experimental results. The frequency of fixation points in each AOI was counted as the feature value, and *K* areas of interest correspond to *K* feature values.

### 3.2. Facial Expression Features

Previous researchers have suggested that children with ASD have a defect in facial expression imitation ability compared with TD children [21]. In the field of computer vision, a FER algorithm could be used to analyze children's facial expression imitation ability, which may be feasible to detect children with ASD. Nevertheless, FER remains a challenging task because the facial expressions of ASD children are complex/ambiguous, usually exhibiting a combination of multiple basic emotions instead of a single emotion; hence, traditional FER cannot obtain optimal performance in analyzing the facial expressions of children with ASD [22]. To address this problem, our previous research on FER based on a convolutional neural network (CNN) and a soft label was used as a reference to detect the facial expression of children [23]. A soft label can annotate multiple labels on a combination of expressions, thus providing a highly intuitive description for complex expression images. First, we used a constructor to obtain a soft label, and a CNN model was trained on the basis of a hard label. Then, the probability distribution of the latent label was fused. Moreover, we trained multiple base classifiers to improve the generalization performance of the ensemble classifier. The framework of FER based on a CNN and a soft label is shown in Figure 3. The expression type that appears in the stimulus is defined as the target expression. The facial expressions of the children were recorded, and then, we counted the frames where the target expression appears in the children's facial expressions in every 40 frames. Lastly, the number of target expressions in every 40 frames was used as a facial expression feature.

### 3.3. EEG Features

In this study, the Emotiv EPOC neuroheadset was used to collect EEG signals. It is composed of 14 data acquisition electrodes (AF3, F7, F3, FC5, T7, P7, O1, O2, P8, T8, FC6, F4, F8, and AF4) and 2 reference electrodes (P3 and P4). The electrode distribution strictly follows the international lead design of 10–20 systems. First, we preprocessed the raw EEG signals to reject the outliers. A low-pass filter was used to reject noise with a frequency larger than 45 Hz, and a high-pass filter was utilized to reject noise less than 0.2 Hz. After filtering, data were divided into effective epochs, and invalid data, such as data with an eye blink, eye movement, and muscle movement, were removed. Then, fast Fourier transform was used to obtain five frequency bands: theta (4–6 Hz), alpha (6–13 Hz), low beta (13–20 Hz), high beta (20–30 Hz), and gamma (30–45 Hz) [24]. The powers of the five frequency bands in an effective epoch were extracted, and a *t*-test was run to explore the differences in EEG in various brain regions of the two groups under distinct frequency bands.

Table 1 outlines the independent sample *t*-test for different groups on the power of each band. The theta band of the two groups showed significant differences in the left frontal lobe (*t* = 5.82, *p* < 0.05), right frontal lobe (*t* = 3.02, *p* < 0.05), right temporal lobe (*t* = 2.91, *p* < 0.05), parietal lobe (*t* = 3.67, *p* < 0.05), and occipital lobe (*t* = 4.72, *p* < 0.05). The power of the theta band of the ASD group was significantly higher than that of the TD group. In line with previous studies, the theta band of the ASD group was significantly different from that of the TD group in frontal, temporal, and occipital lobes [25]. From the physiological perspective, theta waves mainly reflect the emotional experience of individuals, particularly those with ASD. Between the ASD and TD groups, no significant difference in the power of alpha band existed in most brain regions, except the parietal lobe (*t* = 2.40, *p* < 0.05) and occipital lobe (*t* = 2.91, *p* < 0.05). The alpha band mainly reflects the deep relaxation state of the brain, and a minimal difference existed between the two groups. In addition, the low-beta band is related to the capacity for concentration, which is absent in children with ASD. Therefore, the differences in the left frontal lobe (*t* = 2.75, *p* < 0.05), right frontal lobe (*t* = 2.92, *p* < 0.05), parietal lobe (*t* = 2.49, *p* < 0.05), and occipital lobe (*t* = 3.65, *p* < 0.05) of the low-beta band were significant. Furthermore, a significant difference existed in the left frontal lobe (*t* = 2.28, *p* < 0.05) of the gamma band, which is mainly related to the abilities of learning, memory, and information processing. The experimental results showed significant differences in the abilities of learning, memory, and information processing between the two groups.

Table 1 indicates that the EEG power of some brain regions can reflect the ability differences of children with ASD and TD children. Hence, in this study, the power of different brain regions with significant differences was extracted as EEG features to distinguish ASD in TD children. The EEG features extracted are as follows: LF of theta, RF of theta, RT of theta, P of theta, O of theta, P of alpha, O of alpha, LF of low beta, RF of low beta, P of low beta, O of low beta, and LF of gamma.

## 4. Multimodal Data Fusion

Multimodal fusion can combine data from different modalities for analysis. The fusion of multimodal data could provide surplus information and is beneficial to improving the accuracy of the final result [26]. In the previous section, we have introduced the features extracted from various modalities. In this section, we discuss an approach to combining the features to obtain an overall result.

### 4.1. Weighted Naive Bayes Algorithm

To date, three methods for multimodal data fusion exist: feature fusion, decision fusion, and hybrid fusion. For feature fusion, the features extracted from various modalities are fused as a single feature vector, which is analyzed for decision. In decision fusion, the decision results of each modality are fused as a decision vector to gain an overall result. Hybrid fusion will be elaborated in detail in Subsection 4.2. In decision fusion, the features of each modality are independently classified, and the classification results of each modality are identified as subdecisions. To fuse the subdecisions of different modalities and obtain a comprehensive classification result, we adopted a naive Bayes algorithm based on attribute weighting to calculate the weight of the subdecisions [27, 28]. In accordance with the Bayes algorithm, the probability of a child being identified as ASD can be defined as follows:

(5) $$\begin{array}{c} P\left(c_{i}|d_{1},d_{2},\ldots ,d_{n}\right)=\frac{P\left(d_{1},d_{2},\ldots ,d_{n},c_{i}\right)}{P\left(d_{1},d_{2},\ldots ,d_{n}\right)}, \end{array}$$

where *C* is the set of classification results, and *d*_*n*_ represents the subdecisions of different modalities. *P*(*d*_1_, *d*_2_,…, *d*_*n*_, *c*_*i*_) represents the probability that the classification result is *c*_*i*_ under the condition that the subdecision combination is {*d*_1_, *d*_2_,…, *d*_*n*_}. *P*(*d*_1_, *d*_2_,…, *d*_*n*_) is the probability of {*d*_1_, *d*_2_,…, *d*_*n*_} appearing in the training data. The joint probability of *d*_1_, *d*_2_,…, *d*_*n*_ can be expressed as the product of the probabilities of each attribute. Therefore, the probability of a child being identified as ASD can be defined as follows:

(6) $$\begin{array}{c} P\left(c_{i}|d_{1},d_{2},\ldots ,d_{n}\right)=\frac{\prod_{j=1}^{n}P\left(d_{j},c_{i}\right)}{P\left(d_{1},d_{2},\ldots ,d_{n}\right)} \end{array}$$

However, a deviation existed between the calculated and actual results. In formula (6), the naive Bayes algorithm assumes that each attribute has the same influence on the classification result; in fact, they are different. In the process of constructing a naive Bayes classifier, we used a weighting coefficient to represent the influence of each attribute on the classification to improve the classification accuracy. The posterior probability was calculated by weighting the conditional probability of each attribute. The attributes that are highly correlated with the classification results will have a large weighting coefficient and vice versa. The weighting coefficient for each probability *P*(*d*_*m*_=*v|c*_*i*_) can be calculated as follows:

(7) $$\begin{array}{c} W_{\left(d_{m}=v|c_{i}\right)}=\frac{n\left(m\right)+n\left(d_{m}=v\wedge c_{i}\right)/n\left(d_{m}=v\right)}{n\left(m\right)}, \end{array}$$

where *n*(*m*) represents the number of decisions, and *n*(*d*_*m*_=*v*∧*c*_*i*_) represents the number of instances in the training set in which the classification result is *c*_*i*_ and the value of *d*_*m*_ is *v*. *n*(*d*_*m*_=*v*) represents the number of instances in the training set in which *d*_*m*_ is the value of *v*.

In formula (7), the attribute weight can be prevented to be 0. If the number of instances corresponding to *c*_*i*_ is relatively large, the attribute will obtain a large weighted value. The probability of a child being identified as ASD or TD by using the attribute-weighted naive Bayes algorithm can be defined as follows:

(8) $$\begin{array}{c} P\left(c_{i}|d_{1},d_{2},\ldots ,d_{n}\right)=\frac{\prod_{j=1}^{n}P\left(d_{j},c_{i}\right)*W\left(k_{j}|c_{i}\right)}{P\left(d_{1},d_{2},\ldots ,d_{n}\right)}. \end{array}$$

### 4.2. Hybrid Fusion Framework Based on a Weighted Naive Bayes Algorithm

Hybrid fusion is the combination of feature fusion and decision fusion, and it utilizes the merits of feature fusion and decision fusion and overcomes their disadvantages. In this study, we proposed a multimodal framework based on hybrid fusion, as shown in Figure 4.

In the hybrid fusion framework, the features *f*_1_, *f*_2_, and *f*_3_ of EEG, facial expression, and eye fixation were extracted, respectively. *f*_1_ is a physiological feature, whereas *f*_2_ and *f*_3_ are behavioral features. To exploit the correlation of different behavioral features, we performed feature fusion in the early stage. In level 1, facial expression feature vector *f2* and eye fixation feature vector *f*_3_ were combined as a general vector, which was sent for classification with the result of *d*_2_^(1)^. Hence, *d*_1_^(1)^ is the subdecision of the physiological feature, and *d*_2_^(1)^ is the subdecision of the behavioral features. In level 2, *d*_1_^(1)^ and *d*_2_^(1)^ were fused as a decision vector, and decision fusion was used to obtain the final decision *d*^(2)^. A traditional Bayes algorithm assumes that all attributes play the same role in the result. However, in fact, the influence of each attribute on the result is different. This study proposed a weighted naive Bayes algorithm, as described in Subsection 4.1. An attribute with a high correlation will obtain a large weighted coefficient and vice versa. *W*_1_^(1)^ and *W*_2_^(1)^ are the decision weights of *d*_1_^(1)^ and *d*_2_^(1)^, respectively. *P*_1_ is the probability of a child being identified as ASD, whereas *P*_2_ is the probability of a child being identified as TD. The larger probability corresponds to the final prediction result.

## 5. Experiment and Data Analysis

In this study, 80 children, including 40 ASD children and 40 TD children, completed the experimental task, and leave-one-out cross validation was used to ensure that the training samples are sufficient [29].

### 5.1. Accuracies of Different Classification Methods

We evaluated the accuracy of different modalities with various classifiers to investigate which modality is the best to identify children with ASD. Usually, accuracy is the proportion of correctly classified samples to total samples. We selected three commonly used classifiers to perform the classification: (1) random forest (RF); (2) support-vector machine; and (3) *K*-nearest neighbor. We compared the classification accuracy of each classifier on different modalities, as shown in Table 2. The classification result of EEG data with RF was the best with an accuracy of 83.75%, and the average accuracy of EEG data with different classifiers was 74.69%. Regardless of the best or average classification accuracy, it was higher in EEG data than in other single modalities. These results indicated that EEG may be the most discriminative information compared with eye fixation and facial expression data.

In the hybrid fusion framework proposed in Subsection 4.2, physiological and behavioral features were used for classification with three commonly used classifiers, and then, they were fused using a weighted naive Bayes algorithm. As shown in Table 3, the best classification accuracy of hybrid fusion classification based on weighted naive Bayes was 87.50%, the best accuracy of physiological data was 83.75%, and the best accuracy of behavioral data was 85.00%. These results demonstrated the efficiency of hybrid fusion classification based on weighted naive Bayes, and the combination of behavioral and physiological data can improve the classification accuracy.

### 5.2. Complementary Characteristics of Different Data Modalities

For ASD detection, we obtained an average accuracy of 67.50% by using only the data of eye fixation, 71.56% by using only the data of facial expression, and 74.69% by using only the data of EEG. For hybrid fusion based on a weighted naive Bayes algorithm, two stages were considered: (1) feature fusion in level 1 and (2) decision fusion in level 2. For feature fusion, the feature vectors of facial expression and eye fixation were directly concatenated into a larger feature vector as the inputs of the classifier. In the decision fusion stage, decision weight was calculated in accordance with the influence of each attribute on the result. We obtained the best accuracy of 87.50% by using hybrid modality fusion based on a weighted naive Bayes algorithm. This value was significantly greater than that obtained using a single modality, indicating that hybrid fusion can combine the complementary information in each single modality and effectively enhance the performance.

To investigate the complementary characteristics of different data modalities, we analyzed the confusion matrices and graph of eye fixation classification, facial expression classification, EEG classification, and hybrid fusion classification, which could reveal the advantages and weaknesses of each modality. The confusion matrices of each data modality are shown in Figure 5. The confusion graphs of eye fixation and facial expression, eye fixation and EEG, and facial expression and EEG are presented in Figure 6. EEG had the advantage of classifying ASD (90.00%) compared with eye fixation (62.50%) and facial expression (72.50%), facial expression outperformed EEG in recognizing TD (92.50% versus 77.50%), and eye fixation outperformed EEG in recognizing TD (85.00% versus 77.50%). TD was difficult to recognize by using only EEG, and ASD was difficult to recognize by using only eye fixation or facial expression. Previous studies have shown that atypical brain development in children with ASD appears earlier than atypical behavior, and the critical period of early intervention will be missed if the detection is solely based on behavioral features [14]. In this study, we fused physiological and behavioral features to improve detection accuracy.

Moreover, the misclassifications of the three modalities were different. Eye fixation misclassified more ASDs as TDs (37.50%), whereas EEG misclassified more TDs as ASDs (22.50%). These results indicated that eye fixation, facial expression, and EEG had different discriminative powers for ASD and TD recognition, and they presented important complementary characteristics. As shown in Table 3, combining the complementary information of the three modalities, that is, hybrid fusion, can significantly improve the classification accuracy (87.50%).

## 6. Conclusions

Early detection of ASD is highly beneficial to treatment. In this study, we proposed a hybrid fusion approach that fuses data on eye fixation, facial expression, and EEG to detect children with ASD. Its implementation can improve detection efficiency and reduce costs. Our main contributions are threefold. First, we have used a novel combination of eye fixation, facial expression, and EEG data for early ASD detection. Second, we have used an innovative approach to extract features: (1) eye fixation features based on *k*-means algorithm; (2) facial expression features based on a CNN and a soft label; and (3) 12 EEG features based on the power of different brain regions. Third, we have presented a hybrid fusion approach based on a weighted naive Bayes algorithm for multimodal data fusion. Our results indicate that the hybrid fusion classification in this study is efficient for the early detection of ASD. Eye fixation, facial expression, and EEG have different discriminative powers for ASD and TD detection, and EEG may be the most discriminative information compared with eye fixation and facial expression. The three modalities have important complementary characteristics, and hybrid fusion can significantly improve classification accuracy by combining their complementary information.

However, despite our promising findings and their potential application prospect, limitations remain. First, the number of samples used was relatively small. Extending the study to include more subjects could improve the accuracy and stability of the algorithm. In the future, we plan to increase the number of children sampled. Second, the data used have nonstationary characteristics, and the recording environments are changing. Consequently, across-day variability exists in recording conditions. In the future, adopting detection models over time should be further studied.

## Figures and Tables

**Figure 1:** The experimental scene and data analysis framework. *Note.* Data were collected using Tobii Eye Tracker, Emotiv EPOC+, and camera, providing the eye fixation, EEG, and facial expression data, respectively.

**Figure 2:** Different AOI divided by *K*-means algorithm. (a) *K* = 8, (b) *K* = 12, (c) *K* = 16, (d) *K* = 20.

**Figure 3:** The framework of facial expression recognition based on convolutional neural network (CNN) and soft label.

**Figure 4:** Hybrid fusion framework based on weighted naive Bayes algorithm.

**Figure 5:** Confusion matrices of single modality classification and hybrid fusion classification. *Note.* The row of each of the confusion matrices represents the predicted class, and the column represents the target class. The element (*i*, *j*) is the percentage of samples in class *j* that is predicted as class *i.* (a) Eye fixation. (b) Facial expression. (c) EEG. (d) Hybrid fusion based on weighted naive Bayes.

**Figure 6:** Confusion graph of single modality, showing their complementary characteristics for identification ASD and TD. The numbers represent the percentage of samples in the class of arrow tail predicted as the class of head. (a) The complementary characteristics of eye fixation and facial expression. (b) The complementary characteristics of eye fixation and EEG. (c) The complementary characteristics of facial expression and EEG.

**Table 1:** *t*-test on the power of each band in different brain regions of children with ASD and TD.

		*F*	*t*	*p*	Mean difference	Std. error difference
Theta	LF^*∗∗*^	7.38	5.82	0.00	4.55	0.72
	RF^*∗*^	1.85	3.02	0.01	3.46	1.08
	LT	1.80	−0.81	0.42	−0.94	1.07
	RT^*∗*^	13.53	2.91	0.01	3.82	1.20
	P^*∗∗*^	11.47	3.67	0.00	4.16	1.12
	O^*∗∗*^	13.50	4.72	0.00	4.44	0.88

Alpha	LF	0.30	2.01	0.05	1.27	0.63
	RF	0.41	1.77	0.09	1.27	0.73
	LT	0.22	−0.86	0.40	−0.49	0.52
	RT	0.92	1.10	0.28	0.92	0.84
	P^*∗*^	7.52	2.40	0.02	1.85	0.73
	O^*∗*^	5.74	2.91	0.01	1.77	0.58
Low beta	LF^*∗*^	1.31	2.75	0.01	0.86	0.31
	RF^*∗*^	2.90	2.92	0.01	0.95	1.78
	LT	1.33	0.36	0.72	0.18	0.50
	RT	1.25	1.73	0.09	0.83	0.55
	P^*∗*^	9.16	2.49	0.02	1.94	0.75
	O^*∗∗*^	8.48	3.65	0.00	0.87	0.23

High beta	LF	1.16	1.80	0.08	0.75	0.40
	RF	2.63	1.80	0.08	0.83	0.47
	LT	4.17	0.78	0.44	0.73	0.88
	RT	0.06	0.28	0.79	0.25	0.91
	P	5.02	1.59	0.12	1.65	1.00
	O	2.73	1.43	0.16	0.33	0.20

Gamma	LF^*∗*^	5.09	2.28	0.03	1.25	0.55
	RF	3.16	1.77	0.09	1.32	0.74
	LT	0.11	−0.22	0.83	−0.28	1.13
	RT	2.28	−0.91	0.37	−1.16	1.14
	P	3.69	1.43	0.16	0.95	0.62
	O	1.26	1.09	0.28	0.20	0.16

*Note.* LF = Left frontal, RF = right frontal, LT = left temporal, RT = right temporal, P = parietal, O = occipital, AF3, F7, F3, FC5, T7, P7, O1, O2, P8, T8, FC6, F4, F8, and AF4 are 14 channels defined by the international 10–20 system. ^*∗*^*p* < 0.05. ^*∗∗*^*p* < 0.01.

**Table 2:** Accuracies of single modality classification (%).

Classifier	Eye fixation data	Facial expression data	EEG data
RF	73.75	77.50	83.75
SVM	65.00	61.25	65.00
KNN	70.00	65.00	72.50
AVG	67.50	71.56	74.69

*Note.* RF, SVM, and KNN represent decision tree, random forest, support-vector machine, and *K*-nearest neighbor, respectively.

**Table 3:** Accuracies of different classification methods (%).

Data	Accuracies of classification
Physiological data classification	83.75
Behavioral data classification	85.00
Hybrid fusion classification	87.50

## Data Availability

The datasets used and/or analyzed during the current study are available from the corresponding author on reasonable request.
